# Effect of SWOT Analysis Combined with the Medical and Nursing Integration Emergency Nursing Process on Emergency Treatment Efficiency and Prognosis of Patients with Acute Myocardial Infarction

**DOI:** 10.1155/2022/7106617

**Published:** 2022-07-30

**Authors:** Cuihuan Wu, Ling Wu, Pan Jin

**Affiliations:** Department of Cardiology, Union Hospital Tongji Medical College, Hua Zhong University of Science and Technology, Wuhan, Hubei 430000, China

## Abstract

Acute myocardial infarction (AMI) is a common clinical emergency. Effective emergency treatment at the early stage of onset can effectively reduce the mortality rate. Time is the key of emergency treatment, which is directly related to the treatment effect and the prognosis of patients, and clinical intensive nursing intervention for emergency treatment is of great significance in improving the efficiency of emergency treatment and prognosis. In this study, the effects of routine emergency care flow and SWOT analysis combined with medical and nursing integration on emergency treatment efficiency and prognosis of patients with acute myocardial infarction were compared. The results showed that the combined scheme could improve the rescue effect and success rate of patients with acute myocardial infarction, shorten the rescue time, and reduce the mortality and complication rate of myocardial infarction, which provided a new direction for clinical emergency treatment of acute myocardial infarction.

## 1. Introduction

Acute myocardial infarction (AMI) refers to the sudden blockage of coronary vessels, causing myocardial ischemia and necrosis in the corresponding area [1]. The onset of this disease is closely related to factors such as overwork, excitement, excessive drinking, overeating, cold stimulation, and constipation. Patients with AMI present with persistent and severe sternal pain or tightness in the chest, and clinical data show that the comprehensive mortality rate of AMI is close to 20% [2]. Previous studies have suggested that the cooperation of effective medical intervention programs in the rescue process of patients with AMI helps to improve the efficiency of emergency treatment and prognosis [3].

At present, situation analysis and medical and nursing integration are both popular nursing models. Among them, situation analysis method, also known as the SWOT analysis method, is a comprehensive and comprehensive analysis method put forward by a professor of management at the University of San Francisco in the early 1980s [4]. In recent years, the SWOT analysis method has been gradually applied to medical care, playing an important role in optimizing nursing work procedures, improving work efficiency, and reducing work omissions [5]. Medical and nursing integration refers to that doctors and nurses form a relatively fixed diagnosis and treatment team to provide patients with treatment and care in the form of a medical care team [6]. Previous studies have respectively reported the application effects of SWOT analysis method and the integrated medical care process in various diseases, but few studies have analyzed the application value of the combined application of the two methods, and their application in AMI still needs to be studied [7]. In view of this, this study analyzed the impact of the SWOT analysis method combined with the medical and nursing integration emergency care process on the emergency treatment efficiency and prognosis of patients with AMI.

## 2. Information and Methods

### 2.1. General Information

A total of 110 patients with AMI who were admitted to our hospital from March 2020 to March 2022 were selected as the research subjects, including 90 males and 20 females. The patients were aged from 40 to 73 years old, with an average age of (62.41 ± 7.55) years old. According to the difference of intervention methods, the patients were divided into a study group and a control group, with 55 cases in each group. There was no statistically significant difference in the general data between the two groups, and they were comparable (*P* > 0.05), as shown in Table 1. This study was approved by the Medical Ethics Committee and informed consent forms were signed for all patients.

### 2.2. Inclusion Criteria

The inclusion criteria were as follows: ① All patients met the diagnostic criteria for AMI [8]. ② Patients under 80 years of age. ③ Patients who can cooperate well with this study.

### 2.3. Exclusion Criteria

The exclusion criteria were as follows: ① Patients with other types of heart disease or cerebrovascular disease and those with related dysfunction. ②Combined with coagulation disorders. ③ Patients with liver and kidney dysfunction. ④ Those combined with senile dementia and mental disease.

### 2.4. Methodology

Patients in the control group were given the routine emergency care procedures. The patient was admitted to the emergency room by medical staff. The patient's medical history was asked in detail, supplemented by an electrocardiogram. At the same time, oxygen inhalation, blood sample collection, and ECG monitoring were performed. The venous access was established immediately after the diagnosis and the preoperative preparation for PCI was completed, after which the patients was transferred to the catheterization room for surgery.

On the basis of the control group, the study group implemented the SWOT analysis of emergency care combined with medical and nursing integration model. The SWOT analysis was as follows: ① Analysis: Analyzing the advantages of our emergency treatment process, we found that our hospital has complete emergency conditions, with adequate staff, high comprehensive level, and complete emergency treatment facilities. According to the summary of clinical work, the disadvantages of emergency treatment in our hospital were mainly as follows: the hospital is in a busy area, which led to a long time for ambulance reception. Analysis of emergency treatment opportunities: The incidence of AMI increased, and the medical-related awareness of the masses was improved. If the number was more than 120 in time, the treatment opportunities for AMI increased. We summarize the challenges faced by our hospital in the first-aid work of AMI. Specifically, the emergency treatment process at 120 is vulnerable to traffic congestion, thus prolonging the treatment time. Due to the tension of medical staff in emergency departments and the insufficient staffing from time to time, emergency rescue has been challenged. In addition, from the perspective of challenges, the high indicators of tasks assigned by the hospital leadership and the high expectations of patients' families have posed a certain degree of challenges to the medical staff in emergency departments. ② Relevant factors such as advantages, disadvantages, opportunities, and threats are arranged in the matrix and systematic analysis is conducted. ③ Implementation of action plan: based on the advantages of our institute, we strengthened the disinfection, device management, and treatment monitoring of ambulances and emergency rooms, and conducted regular and stratified professional comprehensive training for medical staff, as well as real-time simulation training for the mutual cooperation ability of emergency group workers, so as to continuously sum up experience. We comprehensively analyzed the routes of the urban areas where the hospitals are located and the road conditions at different times and planned the receiving routes of the hospitals according to the comprehensive analysis. The ambulance is equipped with a navigation system to understand the road conditions in a timely manner so as to avoid routes with high traffic volume and people flow as much as possible. The optimization of emergency procedures aims to shorten the rescue time as much as possible. The patients in critical condition were treated directly through the green channel in the hospital and explained in detail to their families for simple education.

After the hospital admission, the patients were treated with the integrated medical and nursing integration first-aid care procedures: ① The integrated model was established. According to the situation of department personnel, several integrated teams composed of one emergency doctor and five nurses were formed. ② After patients are admitted, the pre-diagnosis nurse performs rapid evaluation and triage, and then the doctor conducts the primary diagnosis. The rescue nurse coordinated the whole rescue nursing service. One of the other three nurses was responsible for assisting the examination, monitoring and maintenance of vital signs, and observation of illness records. 1 responsible for the management of venous channel, a variety of pipeline management and medication. One nurse is responsible for communication, recording and transfer. In the early stage, the patient was allowed to stay in bed and assisted to complete basic examinations such as myocardial enzymes and ECG. Low flow oxygen was given for 2–5 L/min. The vital signs of patients were detected by ECG monitoring. Arterial blood was also drawn and blood gas analysis results were monitored. In the middle stage, a venous channel was established for intravenous administration and oral administration of drugs as per doctor's advice. Later stage is the first-aid stage. The rescue nurses assess the risk factors based on the patients' examinations and vital signs, confirm the implementation of doctor's advice, check the examination results, assist the doctors to rescue, and finally escort the patients into the catheter room.

### 2.5. Observation Indicators

The observation indicators were as follows:

1. Comparison of the time of emergency rescue indexes between the two groups in emergencies, including triage evaluation time, ECG reporting time, venous blood collection time, and time from admission to start of PCI.
2. Comparison of the rescue success rate between the two groups.
3. The clinical outcomes of the two groups were compared, including the incidence of symptomatic cerebral hemorrhage and mortality of the patients, as well as the National Institutes of Health Stroke Scale (NIHSS) scores [9] at the time of admission and discharge.
4. Comparison of patients' satisfaction in emergency care between the two groups. Nursing satisfaction was recorded by using the self-made nursing satisfaction questionnaire in our hospital. The full score of the scale was 100, with 90–100 being very satisfactory, 70–89 being satisfactory, 50–69 being general satisfactory and <50 being unsatisfactory. Total satisfaction = (very satisfactory + satisfactory + general satisfactory)/total cases × 100%.
5. The incidence of complications in the two groups was counted, including deep vein thrombosis, pseudoaneurysm, urinary retention, and local hemorrhage. The total incidence of complications was compared between the two groups.

### 2.6. Statistical Methods

SPSS 20.0 statistical software was used for analysis. The measurement data were expressed as ($\bar{x}$ ±S) and *t* test was performed. The count data were expressed as percentage (%) using the *χ*^2^ test, and *P* < 0.05 indicated that the difference was statistically significant.

## 3. Results

### 3.1. Comparison of Emergency Rescue Index Time between the Two Groups

The study components' diagnosis and evaluation time, ECG reporting time, venous blood collection time, and time from admission to start of PCI were all shorter than those in the control group (*P* < 0.05) as shown in Table 2.

### 3.2. Comparison of the Rescue Success Rate between the Two Groups

The success rate of rescue in the research group was higher than that of the control group (*P* < 0.05) as shown in Table 3.

### 3.3. Comparison of Clinical Outcomes between the Two Groups

The incidence and mortality of symptomatic cerebral hemorrhage in the study group were lower than those in the control group (*P* < 0.05). There was no difference in the NHISS score between the two groups on admission (*P* > 0.05), while the NHISS score in the research group was lower than that in the control group after discharge at (*P* < 0.05) as shown in Table 4.

### 3.4. Comparison of Patients' Satisfaction with Emergency Care between the Two Groups

The total satisfaction degree of patients in the research group on emergency care was higher than that in the control group (*P* < 0.05), as shown in Table 5.

### 3.5. Comparison of Complication Rates between the Two Groups

The incidence of complications in the study group was lower than that in the control group (*P* < 0.05) as shown in Table 6.

## 4. Discussion

AMI is characterized by acute onset and high mortality. The key to treatment is to open the infarct vessel as early as possible in the early stage of onset, to save the frequently died myocardium and to prevent the infarct size from expanding [10]. Research has shown that treatment with timely and effective nursing measures can improve the success rate of clinical rescue and improve the prognosis [11]. Therefore, the establishment of efficient emergency treatment mode has long been the focus of exploration and efforts of health care workers.

This study showed that the durations of emergency rescue indexes in the study group were shorter than those in the control group, and the success rate of emergency rescue in the research group was higher than that in the control group (*P* < 0.05). These results indicated that the combined use of the SWOT analysis method and the medical and nursing integration emergency care process were conducive to reducing the retention time of patients before PCI, effectively shortening the overall treatment time, speeding up the recovery of myocardial blood supply, and improving the rescue efficiency of patients with AMI. The SWOT analysis method is an analysis method that measures the internal competitive environment and competitive conditions of the organization, analyzes the advantages and disadvantages and identifies the challenges faced by the related work, and further formulates and implements the solution according to the specific analysis results, so that the related work can be effectively solved. [12]. The study believed that introducing it into nursing management could objectively and comprehensively analyze the internal and external environment of nursing organization, formulate scientific nursing countermeasures according to the constructed situation matrix, and enhance the scientificity of nursing management and the market adaptability of nursing organization [13]. In this study, SWOT analysis has two functions in emergency nursing. On the one hand, the implementation of SWOT analysis comprehensively summarizes the advantages and disadvantages of emergency science and technology, emergency procedures and emergency work in our hospital, and provides a scientific basis for the planning of emergency procedures. On the other hand, at the same time, through a series of measures such as strengthening the quality supervision of ambulances and emergency rooms, strengthening the comprehensive training of medical staff in departments, optimizing the emergency receiving route and treatment process, it helps the emergency department to make full use of our hospital's high-quality emergency treatment conditions and facilities. It greatly improved the quality of AMI emergency care, improve the efficiency of emergency treatment, enhance the effect of treatment, and improve the prognosis of patients [14, 15].

As recommended in the guidelines of the Global Definition of Myocardial Infarction, the patient presented with a balloon dilatation time of less than 90 min, in order to obtain maximum reperfusion [16]. Therefore, the nursing process is also a very important part in the emergency treatment process [17]. The high-quality and efficient emergency nursing process is one of the important guarantees for improving the survival rate of patients with AMI [18]. This study focused on optimizing and improving the emergency process of AMI patients in the emergency department under the SWOT analysis method and applied the medical and nursing integration intervention model to the emergency care process. Moreover, the result showed that the incidence rate and mortality rate of symptomatic cerebral hemorrhage in the study group were lower than those in the control group (*P* < 0.05), which further confirmed that the combination of the SWOT analysis method and emergency medical care process could optimize the emergency procedures of AMI, reduce the incidence and mortality rate of complications such as symptomatic cerebral hemorrhage, and improve the prognosis of patients. First of all, an integrated team composed of one emergency doctor and five nurses was formed to clarify the work content of each person. Meanwhile, the medical care, nursing care, and patient care were integrated into the emergency work through the procedures [18]. The procedures were improved so as to strengthen the cooperation between medical care and avoid the problems such as unclear responsibilities, unclear responsibilities, unclear handover, nursing interruption, and nursing gap from delaying the treatment [19]. In addition, the medical and nursing integration emergency first-aid care process can ensure that the dying myocardial cells are saved in the shortest time, thereby improving the success rate of rescue and reducing the occurrence of complications, death, and relapse [20].

In addition, this study showed that the total satisfaction of patients in the study group on emergency care was higher than that in the control group (*P* < 0.05), indicating that the implementation of this model helped to narrow the relationship between nurses and patients. The reason was that while implementing the SWOT analysis method and the medical integrated emergency care process, the medical staff also effectively managed the emotions and cognition of the family members, thus improving their understanding of and support for the nursing work [21, 22].

In summary, the implementation of the SWOT analysis method combined with the medical and nursing integration emergency care process can improve the rescue effect and the success rate of rescue of patients with AMI, shorten the rescue time, and reduce the mortality rate and the incidence of complications, which is worthy of clinical application. The shortcoming of this study lies in that the included sample size is only 110, and the sample size can be expanded in the future to further verify the impact of the SWOT analysis method combined with the medical and nursing integration emergency care process on patients with acute myocardial infarction.

## Figures and Tables

**Table 1:** Comparison of general data of patients between the two groups.

Group	n	*Gender (n)*		Age (years old)	BMI (kg/㎡)	*Types of infarction (n)*			
		Male	Female			Anterior wall and anterior septal wall infarction	Extensive anterior wall infarction	Inferior wall and inferior lateral wall infarction	High lateral wall infarction
Study group	55	48	7	62.54 ± 7.26	24.71 ± 2.74	17	13	10	15
Control group	55	42	13	62.62 ± 7.31	24.63 ± 2.33	15	14	12	14
*χ* ^2^/*t*	—	2.200	0.058	0.165		0.378			
*P*	—	0.138	0.954	0.869		0.945			

**Table 2:** Comparison of emergency rescue index time between the two groups (min, $\bar{x}$ ±S).

Group	n	Triage evaluation time	ECG reporting time	Venous blood collection time	Time from admission to start of PCI
Study group	55	1.43 ± 0.52	4.25 ± 1.24	4.89 ± 1.37	6.95 ± 1.24
Control group	55	2.17 ± 0.49	5.79 ± 1.57	6.96 ± 1.48	14.53 ± 1.69
*T*	—	7.681	5.709	7.612	26.819
*P*	—	<0.001	<0.001	<0.001	<0.001

**Table 3:** Comparison of the rescue success rate between the two groups (n, %).

Group	N	Number of cases	Percentage
Study group	55	51	92.73
Control group	55	43	78.18
*t*	—	4.681	
*P*	—	0.031	

**Table 4:** Comparison of clinical outcomes between the two groups.

Group	N	NHISS (score)		Symptomatic cerebral hemorrhage (n, %)	Mortality (n, %)
		On admission	After discharge		
Study group	55	19.69 ± 4.52	7.15 ± 2.23^a^	1 (1.82)	4 (7.25)
Control group	55	19.48 ± 4.36	9.46 ± 1.69^a^	7 (12.73)	13 (23.64)
*χ* ^2^/*t*	—	0.248	6.123	4.853	5.636
*P*	—	0.805	<0.001	0.028	0.018

Compared to the time of admission, ^a^*P* < 0.05.

**Table 5:** Comparison of patients' satisfaction with emergency care between the two groups (n, %).

Group	n	Very satisfactory	Satisfactory	General satisfactory	Unsatisfactory	Total satisfaction
Study group	55	31 (56.36)	12 (21.82)	10 (18.18)	2 (3.64)	53 (96.36)
Control group	55	24 (43.64)	15 (27.27)	7 (12.73)	9 (16.36)	46 (83.64)
*χ* ^2^	—					4.949
*P*	—					0.026

**Table 6:** Comparison of complications between the two groups (n, %).

Group	n	Deep vein thrombosis	Pseudoaneurysm	Urinary retention	Local hemorrhage	Total incidence
Study group	55	0 (0.00)	1 (1.82)	1 (1.82)	0 (0.00)	2 (3.64)
Control group	55	2 (3.64)	4 (7.27)	2 (3.64)	1 (2.82)	9 (16.36)
*χ* ^2^	—					4.949
*P*	—					0.026

## Data Availability

The data used and/or analyzed during the current study are available from the corresponding author upon request.
